# The clinical value of the hepatic venous pressure gradient in patients undergoing hepatic resection for hepatocellular carcinoma with or without liver cirrhosis

**DOI:** 10.1515/med-2023-0851

**Published:** 2024-03-08

**Authors:** Felix Busch, Katja N. De Paepe, Paul Gibbs, Michael Allison, Matthew Hoare, Teik Choon See

**Affiliations:** Department of Radiology, Charité – Universitätsmedizin Berlin, Hindenburgdamm 30, Berlin, 12203, Germany; Department of Radiology, Cambridge University Hospitals NHS Foundation Trust, Addenbrooke's Hospital, Cambridge, CB2 0QQ, United Kingdom; Department of Surgery, Cambridge University Hospitals NHS Foundation Trust, Addenbrooke's Hospital, Cambridge, CB2 0QQ, United Kingdom; Department of Hepatology, Cambridge University Hospitals NHS Foundation Trust, Addenbrooke's Hospital, Cambridge, CB2 0QQ, United Kingdom; Early Cancer Institute, University of Cambridge, Hutchison Research Institute, Cambridge, CB2 0XZ, United Kingdom

**Keywords:** hepatic venous pressure gradient measurement, HCC, advanced chronic liver disease, liver resection, clinically significant portal hypertension

## Abstract

The role of hepatic venous pressure gradient (HVPG) measurement in risk stratification before liver resection is an ongoing area of debate. This study examines the impact of preoperative HVPG levels on overall survival (OS)/time to recurrence (TTR) and postoperative complications after hepatic resection of hepatocellular carcinoma (HCC). Thirty-eight HCC patients undergoing HVPG measurement before liver resection at Cambridge University Hospitals NHS Foundation Trust between January 2014 and April 2022 were retrospectively analysed. Statistical analysis comprised univariable/multivariable Cox/logistic regression to identify risk factors of reduced OS/TTR or 90-day post-resection complications and Kaplan–Meier estimator, log-rank, chi-squared, Fisher's exact, and Mann–Whitney *U* test, or Student's *t*-test for survival/subgroup analysis. The median HPVG was 6 (range: 0–14) mmHg. The HVPG was an independent risk factor for poorer TTR in the overall cohort (cut-off: ≥7.5 mmHg (17.18/43.81 months; *P* = 0.009)). In the subgroup analysis of cirrhotic patients (*N* = 29 (76%)), HVPG was additionally an independent risk factor for lower OS (cut-off: ≥8.5 mmHg [44.39/76.84 months; *P* = 0.012]). The HVPG had no impact on OS/TTR in non-cirrhotic patients (*N* = 9 (24%)), nor was it associated with postoperative complications in any cohort. In conclusion, preoperative HVPG levels are useful predictors for TTR and OS in cirrhotic HCC patients undergoing hepatic resection.

## 1 Introduction

Advanced chronic liver disease usually leads to increased portal venous pressure due to fibrotic progression of the liver parenchyma, which is associated with life-threatening complications, such as variceal haemorrhage, hepatorenal syndrome, or hepatic encephalopathy [1,2]. The assessment of portal venous pressure is known to be a useful tool for monitoring disease progress and treatment response in patients with chronic liver disease [3].

The hepatic venous pressure gradient (HVPG) measurement is an invasive although safe method for a precise indirect estimation of the portal venous pressure and has therefore become the standard measurement method in recent decades [3,4]. HVPG values of 5–9 mmHg are considered mild portal hypertension and, e.g., are associated with a higher risk of HCV recurrence after liver transplantation [5,6]. Values ≥10 mmHg are categorised as clinically significant portal hypertension (CSPH) and have been linked to the development of hepatocellular carcinoma (HCC), a higher risk of ascites, variceal bleeding, or hepatic encephalopathy in patients with compensated cirrhosis [7,8,9]. A meta-analysis in 2015 of eleven studies with a total of 1,737 included subjects concluded a decreased 3- and 5-year overall survival (OS) in HCC patients with compensated cirrhosis and pre-surgical CSPH as well as an increased risk of liver decompensation in a sub-analysis after liver resection of HCC [10]. However, in this pooled analysis, patients with CSPH had significantly higher bilirubin levels and a higher international normalised ratio and were more often Child-Pugh class B at baseline than non-CSPH patients [11]. In a propensity score matching study, patients with portal hypertension (indirectly assessed by reduced platelet count and splenomegaly or the presence of gastroesophageal varices) with the same model for end-stage liver disease (MELD) score and extent of hepatectomy planning showed no inferior survival or a higher number of postoperative complications [12]. A recent study showed safe postoperative courses and promising 5-year OS and disease-free survival rates of 55 and 43%, respectively, after liver resection of HCC in Child-Pugh A patients with CSPH [13]. In addition, it has been reported that one-quarter of HCC patients who would benefit from surgery are excluded when CSPH is considered a contraindication [14].

Hence, there is an ongoing discourse about the impact of increased preoperative HVPG levels, especially when amounting to CSPH, on postoperative complications and the long-term outcome in HCC patients undergoing liver resection. Moreover, the current literature is still based on small sample sizes, and international guidelines do not recommend the HVPG measurement before resection per se due to the minimally invasive procedure, cost-intensiveness, and the requirement of interventional expertise that is usually only available in large tertiary centres [13,15,16,17]. Finally, no study has separately investigated the impact of HVPG levels on post-resection complications or the long-term outcome for non-cirrhotic patients with HCC.

Therefore, the purpose of this study is to investigate the value of HVPG measurements prior to liver resection in HCC patients with or without cirrhosis, determining the impact of the pre-resection HVPG level on OS, time to recurrence (TTR), 90-day post-resection complications, and hospital length of stay after liver resection of HCC with curative intent.

## 2 Methods

Institutional approval was obtained for this retrospective study (PRN10518). All subjects gave informed consent prior to HVPG measurement.

### 2.1 Inclusion and exclusion criteria

This study included patients ≥18 years of age with histologically or radiologically (Liver Imaging Reporting And Data System 5) diagnosed HCC who underwent HVPG measurement prior to liver resection with curative intent at Cambridge University Hospitals NHS Foundation Trust, UK, between January 2014 and April 2022 [18]. Patients with a previous liver resection at the same lesion site or those ultimately not undergoing liver resection after HVPG assessment were excluded from the analysis.

### 2.2 Study endpoints and parameters

The primary endpoint was to evaluate the impact of the pre-resection HVPG level on OS, TTR, the development of 90-day post-resection complications, and post-resection hospital stay length in HCC patients undergoing liver resection with or without liver cirrhosis. In a subgroup analysis, we compared the same endpoints between patients with and without preoperative CSPH (HVPG values ≥10 mmHg) independently of present cirrhosis. The presence of liver cirrhosis was determined from the pathological reports of liver resection. OS was defined as the time from curative resection to death. TTR was defined as the time from resection to progression of intra- or extrahepatic HCC disease, censoring death without recurrence at the time of death.

In addition, all other obtained basic and disease-specific patient characteristics at baseline were examined on their effect on OS, TTR, 90-day post-resection complications, and hospital stay length (see Table 1). Ascites was graded according to the Consensus Conference of the International Ascites Club [19]. Splenomegaly was defined as a major diameter >10 cm on axial CT or MRI [20]. Additionally included surgical parameters were resection approach, resection extent (minor resection of up to two or major resection of more than two liver segments [21]), and anatomical/non-anatomical resection.

**Table 1:** Preoperative basic and disease characteristics of the overall cohort and the comparison of patients with/without cirrhosis and patients with/without clinically significant portal hypertension (≥10 mmHg)

Variables	Overall cohort (*N* = 38)	Cirrhosis (*N* = 29)	Non-cirrhotic (*N* = 9)	*P* value comparison	HVPG ≥10 mmHg (*N* = 10)	HVPG <10 mmHg (*N* = 28)	*P* value comparison
Age (years)	66 (40–77)	66 (40–76)	66 (56–77)	0.480	57 (52–72)	66 (40–77)	0.183
Sex (*N*)				0.396			0.090
Female	10	9	1		5	5	
Male	28	20	8		5	23	
Body mass index (kg/m^2^)*	28.16 ± 4.92	27.54 ± 4.89	29.97 ± 4.81	0.206	28.12 ± 5	28.17 ± 4.99	0.979
Extrahepatic disease (*N*)				1.000			1.000
Bladder cancer	1	1	0		0	1	
Number of lesions (*N*)	1 (1–4)	1 (1–4)	1 (1–2)	1.000	1 (1–3)	1 (1–4)	0.097
Median lesion size (mm)	30 (9.5–110)	25 (9.5–82)	37 (17–110)	0.050	16 (9.5–34.67)	32.75 (11–110)	**0.029**
Size of largest lesion (mm)	30 (12–110)	25 (12–79)	55 (17–110)	**0.004**	21 (13–64)	33.5 (12–110)	0.445
UICC staging 8th edition (*N*)				0.557			0.135
pT1 a/b	5/2	4/2	1/0		2/2	3/0	
pT2	20	16	4		6	14	
pT3	5	4	1		0	5	
pT4	5	2	3		0	5	
pTx	1	1	0		0	1	
R1	6	5	1		0	6	
Histological grading (*N*)				0.164			0.218
G1	7	5	2		4	3	
G2	19	17	2		4	15	
G3	11	6	5		2	9	
GX	1	1	0		0	1	
Microscopic vascular invasion (*N*)	27	19	8	0.237	5	22	0.236
Macroscopic vascular invasion (*N*)	10	4	6	**0.005**	1	9	0.116
HCC aetiology (*N*)				0.239			0.768
Hepatitis C virus	17	11	6		4	13	
Hepatitis B virus	2	0	1		1	1	
Non-alcoholic fatty liver disease	11	9	2		2	9	
Alcohol abuse	3	3	0		1	2	
Primary biliary cholangitis	4	4	0		2	2	
Cryptogenic	1	0	1		0	1	
Alpha fetoprotein (kU/L)	11 (0–30,335)	8.5 (0–30,335)	30 (1–23,106)	0.154	12 (4–2,345)	10 (0–30,335)	0.496
Albumin (g/L)*	36.39 ± 4.33	36.38 ± 4.68	36.44 ± 3.21	0.969	34 ± 3.2	37.25 ± 4.41	**0.040**
Serum creatinine (μmol/L)	70 (48–129)	72.5 (48–129)	70 (48–127)	0.757	59 (48–129)	76 (48–127)	**0.037**
Total bilirubin (μmol/L)	10 (6–24)	11.5 (7–24)	8 (6–14)	**0.027**	11 (7–24)	10 (6–20)	0.198
INR	1.09 (0.87–1.89)	1.1 (0.96–1.89)	1.07 (0.87–1.25)	0.302	1.09 (0.96–1.34)	1.07 (0.87–1.89)	0.842
Serum sodium (mmol/L)	139 (123–143)	139 (123–143)	139 (137–140)	0.519	139 (136–141)	138.5 (123–143)	0.590
Platelet count (×10^3^/mm^3^)*	179.16 ± 61.57	165 ± 58.95	224.78 ± 47.98	**0.009**	141.3 ± 54.25	192.68 ± 59.11	**0.021**
ECOG performance status (*N*)				0.297			0.610
0	30	21	9		8	22	
1	5	5	0		2	3	
Not applicable	3	3	0		0	3	
Child-Pugh class (*N*)				1.000			0.462
A	36	27	9		9	27	
B	2	2	0		1	1	
BCLC stage (*N*)				0.472			0.575
0	2	2	0		1	1	
A	31	22	9		8	23	
B	2	2	0		1	1	
Not applicable	3	3	0		0	3	
MELD score	7 (6–24)	8 (6–24)	7 (6–11)	0.471	7 (6–10)	6 (6–24)	0.351
Wedged hepatic venous pressure (mmHg)	17.25 (7.5–35)	17 (8–34.5)	18 (7.5–35)	0.948	22.67 (14.5–23.67)	17 (7.5–35)	0.068
Free hepatic venous pressure (mmHg)	10.84 (3–27.33)	10.67 (3–26.67)	11.5 (6.5–27.33)	0.429	9.5 (3–13.5)	11 (4–27.33)	0.507
HVPG (mmHg)	6 (0–14)	6 (2–14)	5 (0–11)	0.110	11.17 (10.17–14)	5 (0–9)	**<0.001**
HVPG 5–9 mmHg (*N*)	17	13	4	1.000	0	17	**<0.001**
HVPG ≥10 mmHg (*N*)	10	9	1	0.396	10	0	**<0.001**
Inferior vena cava pressure (mmHg)	10 (2–28)	10 (2–24)	10 (5–28)	0.739	8 (3–13)	10 (2–28)	0.578
Right atrial pressure (mmHg)	6.5 (−3–23)	6 (−3–23)	7 (0–22)	0.420	4 (−1–9)	7 (−3–23)	0.369
Diabetes mellitus (*N*)	8	6	2	1.000	0	8	0.082
Arterial hypertension (*N*)	16	11	5	0.450	2	14	0.143
COPD (*N*)	2	2	0	1.000	0	2	1.000
Cirrhosis (*N*)				**<0.001**			0.396
Compensated	28	28	0		8	20	
Decompensated (only grade 1 ascites)	1	1	0		1	0	
Pathological grading background liver (*N*)				**<0.001**			0.497
Healthy	3	0	3		0	3	
Bridging fibrosis	5	0	5		1	4	
Moderate fibrosis	1	0	1		0	1	
Established cirrhosis	18	18	0		7	11	
Complete cirrhosis	11	11	0		2	9	
Splenomegaly (*N*)	2	2	0	1.000	1	1	0.462
Gastroesophageal varices (*N*)	5	5	0	0.312	1	4	1.000
Ascites (*N*)				1.000			0.263
Grade 1	1	1	0		1	0	

Abbreviations: BCLC, Barcelona Clinic Liver Cancer; COPD, chronic obstructive pulmonary disease; ECOG, Eastern Cooperative Oncology Group; HCC, hepatocellular carcinoma; INR, international normalised ratio; HVPG, hepatic venous pressure gradient; MELD, model for end-stage liver disease; UICC, Union for International Cancer Control. *Normally distributed variable displayed with mean ± standard deviation.

Bold values indicate a *P* value < 0.05.

Post-resection complications were analysed for the time of hospitalisation or up to 90 days after resection. Analysed liver complications included liver dysfunction, new or worsening ascites, biliary leakage, hepatic encephalopathy, and post-hepatectomy haemorrhage. Liver dysfunction was defined by 50–50 criteria positive on two or more consecutive days after liver resection, i.e., a prothrombin time of <50% and a serum bilirubin level of >50 µmol/L, considering the blood count on the third, fifth, and seventh days after resection [22,23]. Post-hepatectomy haemorrhage was defined as bleeding requiring transfusion of packed red blood cells for a significant drop in haemoglobin, radiological intervention, or relook laparotomy [24].

Non-liver complications included acute kidney injury, mechanic ileus, pneumonia, type 1 respiratory failure, cardiovascular complications, or sepsis. Prolonged hospitalisation was considered if the hospital stay length exceeded the median of the overall cohort.

### 2.3 HVPG measurement

Potential candidates for HCC resection with clinical or imaging signs suggestive of cirrhosis were referred for HVPG measurement and, if applicable, simultaneous transjugular liver biopsy to assess the severity of advanced chronic liver disease and evaluate the feasibility and safety of liver resection. Measurements were performed by seven consultant interventional radiologists with 2–17 years of experience. Under aseptic technique and local anaesthesia, a 19-G needle was used to puncture the right internal jugular vein (left if the right side is not suitable) under ultrasound guidance. A 7 Fr Super Arrow-Flex® sheath (Teleflex Medical Europe Ltd, Athlon, Leinster, Ireland) was introduced using Seldinger technique, after which a 4 Fr Cobra Catheter (Cordis Corp., Miami Lakes, Florida, USA) was used to cannulate the right or middle hepatic veins. Measurements were performed either with:

(1) A 4 Fr Cobra catheter. The free hepatic venous pressure (FHVP) was measured while the catheter floated freely in the hepatic vein. The wedged hepatic venous pressure (WHVP) was obtained with the catheter wedged into the most distal aspect of the vein until no blood could be aspirated. A wedged venography was performed to confirm the position.
(2) An occlusion balloon catheter (Berenstein, Boston Scientific, Marlborough, Massachusetts, USA). The WHVP was obtained while the inflated balloon occluded the vein. The measured values were retrieved by connecting the catheter to a pressure transducer and monitor. A minimum of three readings were obtained for FHVP and WHVP, respectively. The HVPG was calculated by the difference between the mean WHVP and FHVP of all subsequent measurements. In addition, pressures in the right atrium and inferior vena cava were documented. Patients were monitored and required bed rest for 2 h after the procedure.

### 2.4 Statistical analysis

Statistical analysis was performed using SPSS Statistics 25 (IBM, Armonk, New York, USA). Categorical/nominal variables were reported as frequencies and continuous variables using mean and standard deviation if normally distributed or median and range for non-normally distributed values. Normal distribution was tested with the Shapiro–Wilk test. Univariable/multivariable backward Cox and binary logistic regression were performed to identify risk factors of poorer OS or TTR and 90-day post-resection complications or prolonged hospital stay, respectively. Variables with a *P* value of <0.1 in the univariable analysis were included in multivariable regression analysis to identify independent risk factors. Multicollinearity between variables was tested with Pearson's (if continuous variables) or Spearman's (if categorical/nominal data) correlation analysis (thresholds: ≥0.8/≤−0.8) [25]. Cut-off points were established with the area under receiver operating characteristic curve, choosing the value that maximises the sum of sensitivity and specificity. Kaplan–Meier analysis and log-rank test were used to compare OS and TTR between the determined thresholds and sub-cohorts. The mean survival times with 95% confidence intervals (CI) were reported for better comparability because the median could not be estimated in Kaplan–Meier analysis for all sub-cohorts due to the partially small number of events. Comparison of variables between patients with or without cirrhosis and patients with or without CSPH was performed using the chi-squared test, Fisher's exact test, Mann–Whitney *U* test, or Student's *t*-test, as appropriate. A two-sided asymptotic *P* value of <0.05 was considered significant.

## 3 Results

### 3.1 Study cohort

HPVG measurements for evaluation of HCC resection were performed in 66 patients between January 2014 and April 2022. Twenty-eight (42%) patients were deemed ineligible for resection due to CSPH (*N* = 17 (26%), with HVPG measurements of 12–24 mmHg), insufficient predicted residual liver volume (*N* = 5 (8%)), poor general health condition/HCC involvement of the portal vein (*N* = 2 (3%) each), or hilar lymph node metastases/no further treatment was desired (*N* = 1 (1%) each).

Ultimately, 38 (58%) patients were included for analysis. The median follow-up time was 34.5 (range: 2–81) months. Among the included patients, 10 (26%) patients died (seven (18%) due to HCC recurrence, 3 (8%) due to postoperative complications as below), and 23 (61%) patients developed disease progression during follow-up. The mean OS was 60.36 [95% CI, 49.96–70.76] months and mean TTR 29.4 [95% CI, 19.55–39.25] months. Liver cirrhosis was present in 29 (76%) patients at the time of resection, according to the pathologic reports of liver resection tissue. Three (8%) of the nine (24%) remaining patients had healthy liver background parenchyma, five (13%) bridging fibrosis, and one (3%) moderate fibrosis.

Size of largest lesion, macroscopic vascular invasion, and platelet count were significantly higher in patients with non-cirrhotic HCC, while the total bilirubin level was significantly higher in patients with cirrhosis at baseline. The mean OS for cirrhotic patients (62.27 [95% CI, 50.98–73.56] months) did not differ significantly compared to non-cirrhotic patients (39.4 [95% CI, 28.22–50.58] months; *P* = 0.439). The mean TTR was significantly higher in patients with cirrhosis (34.36 [95% CI, 22.69–46.04] months versus 12.42 [95% CI, 3.41–21.44] months in non-cirrhotic patients; *P* = 0.006). All baseline characteristics of each cohort are displayed in Table 1.

### 3.2 HVPG measurement and treatment characteristics

Table 2 displays all treatment characteristics and observed complications within 90 days after resection.

**Table 2:** Treatment characteristics observed 90-day complications, and postoperative outcome of the overall cohort and the comparison of patients with/without cirrhosis and patients with/without clinically significant portal hypertension (≥10 mmHg)

Variables	Overall cohort (*N* = 38)	Cirrhosis (*N* = 29)	Non-cirrhotic (*N* = 9)	*P* value comparison	HVPG ≥10 mmHg (*N* = 10)	HVPG <10 mmHg (*N* = 28)	*P* value comparison
Pre-HVPG exam therapies (*N*)				0.576			0.773
Radiofrequency ablation	1	1	0		0	1	
Liver resection	1	0	1		0	1	
Transarterial radioembolisation	5	4	1		2	3	
Post-HVPG exam therapies (*N*)				0.507			**0.036**
Resection	38	29	9		10	28	
Radiofrequency ablation	7	5	2		2	5	
Transarterial radioembolisation	11	8	3		4	7	
Re-resection	1	1	0		0		
Liver transplantation	3	3	0		2	1	
Atezolizumab and cabozantinib	1	1	0		1	0	
Atezolizumab and bevacizumab	1	1	0		0	1	
External beam radiotherapy	1	0	1		0	1	
Sorafenib	1	0	1		0	1	
Resection characteristics (*N*)							
Open	38	29	9	1.000	10	28	1.000
Anatomical	6	5	8	1.000	0	6	0.168
Non-anatomical	32	24	1		10	22	
Major (>2 segments)	13	8	5	0.226	2	11	0.441
Minor (1–2 segments)	25	21	4		8	17	
Lengths hospital stay (days)	9 (4–58)	9 (4–58)	7 (4–35)	0.469	8 (4–20)	9 (4–58)	0.527
Complications until 90 days after resection (*N*)							
90-day mortality	3	2	1	1.000	1	2	1.000
Liver dysfunction	5	4	1	1.000	3	2	0.103
Postoperative haemorrhage	4	3	1	1.000	1	3	1.000
Sepsis	2	1	1	0.422	0	2	1.000
New/worsening ascites				0.423			0.685
Grade 1	3	2	1		1	2	
Grade 2	8	6	2		1	7	
Grade 3	1	0	1		0	1	
Hospital-acquired pneumonia	5	5	0	0.312	2	3	0.592
Type 1 respiratory failure	2	2	0	1.000	0	2	1.000
Acute kidney injury	7	6	1	1.000	3	4	0.351
Mechanic ileus	3	3	0	1.000	0	3	0.552
Portal vein thrombosis	1	1	0	1.000	0	1	1.000
Hepatic encephalopathy	1	1	0	1.000	0	1	1.000
Follow-up time (months)	34.5 (2–81)	35 (2–81)	30 (3–51)	0.525	37.5 (11–69)	30 (2–81)	0.426
Disease recurrence (*N*)	23	16	7	**0.006**	9	14	**0.048**
(First) intrahepatic	23	16	7		9	14	
1-year recurrence-free rate	68.9%	77.5%	40%		60%	72.1%	
3-year recurrence-free rate	27.9%	35.8%	0%		0%	42.2%	
Death (*N*)	10	7	3	0.439	5	5	0.146
1-year OS rate	92%	92.8%	88.9%		90%	92.9%	
3-year OS rate	73.6%	77.3%	62.2%		58.3%	82.1%	

Abbreviations: HVPG, hepatic venous pressure gradient; OS, overall survival.

Bold values indicate a *P* value < 0.05.

HVPG measurements were performed with a balloon occlusion (*N* = 4 (11%)) or a Cobra catheter (*N* = 3 (8%)). However, in most patients (*N* = 31 (82%)), it could not be retrospectively determined which of the two catheters was used due to missing information in the interventional reports. The median HVPG was 6 (range: 0–14) mmHg in the overall cohort. Ten (26%) patients had CSPH and 28 (74%) patients HVPG levels <10 mmHg. Patients with CSPH had a significantly lower median lesion size (16 (range: 9.5–34.67) mm versus 32.75 (range: 11–110) mm in non-CSPH patients; *P* = 0.029), serum creatinine levels (59 (range: 48–129) μmol/L versus 76 (range: 48–127) μmol/L; *P* = 0.037), average platelet count (141.3 ± 54.25 ×10^3^/mm^3^ versus 192.68 ± 59.11×10^3^/mm^3^ in non-CSPH patients, *P* = 0.021), and serum albumin levels (34 ± 3.2 g/L versus 37.25 ± 4.41 g/L in non-CSPH patients; *P* = 0.040) at the time of HVPG measurement (Table 1). Post-resection treatments also differed significantly between both groups (see Table 2). Nine (24%) of the ten (26%) patients with CSPH had cirrhosis and one (3%) bridging fibrosis at resection. The measured HVPG in cirrhotic patients was not significantly higher compared to non-cirrhotic patients (6 (range: 2–14) mmHg versus 5 (range: 0–11) mmHg; *P* = 0.110).

Three (8%) patients died within 90 days post-resection after a median time of 35 (range: 20–45) days. Two (5%) patients with HPVG values <5 mmHg died of postoperative pneumonia-associated complications. The third (3%) patient with an HPVG of 14 mmHg died of cardiovascular complications after acute kidney failure and acute coronary syndrome. Liver dysfunction was noted in all three patients who died within 90 days after surgery and in five patients (13%) in total (median HVPG: 11.17, range: 0–13.5 mmHg). Any recorded post-resection complication or the length of hospital admission did not differ between patients with and without cirrhosis or patients with and without CSPH (see Table 2).

### 3.3 Independent risk factors for reduced 90-day survival, OS, and TTR

Cox regression results for 90-day survival, OS, and TTR are shown in Table 3.

**Table 3:** Results of univariable and multivariable Cox regression analysis for 90-day survival, overall survival, and time to recurrence in the overall cohort and patients with or without cirrhosis

Variables	Univariable Cox regression HR (95% CI)	*P* value	Multivariable Cox regression HR (95% CI)	*P* value
**90-day survival in the overall cohort (** ***N*** **= 38)**				
	No variables with *P* < 0.1			
**Overall survival in the overall cohort (** ***N*** **= 38)**				
Age	1.08 (0.99–1.12)	0.075		
**Time to recurrence in the overall cohort (** ***N*** **= 38)**				
HVPG	1.16 (1.02–1.32)	**0.026**	1.26 (1.09–1.46)	**0.002**
Serum creatinine	1.03 (1.00–1.05)	0.071	1.04 (1.02–1.07)	**0.002**
Size of largest lesion	1.02 (0.99–1.04)	0.063	1.03 (1.01–1.05)	**0.004**
**90-day survival in patients with cirrhosis (** ***N*** **= 29)**				
	No variables with *P* < 0.1			
**Overall survival in patients with cirrhosis (** ***N*** **= 29)**				
HVPG	1.28 (1.01–1.61)	**0.041**	1.28 (1.01–1.61)	**0.041**
Total bilirubin	1.14 (0.98–1.33)	0.097		
**Time to recurrence in patients with cirrhosis (** ***N*** **= 29)**				
HVPG	1.26 (1.07–1.50)	**0.007**	1.46 (1.14–1.86)	**0.002**
Serum creatinine	1.05 (1.01–1.10)	**0.009**	1.08 (1.03–1.14)	**0.004**
ECOG status	3.01 (0.87–10.42)	0.082	4.16 (1.00–17.28)	**0.049**
Child-Pugh score	2.00 (1.11–3.60)	**0.020**		
**90-day survival in non-cirrhotic patients (** ***N*** **= 9)**				
	No variables with *P* < 0.1			
**Overall survival in non-cirrhotic patients (** ***N*** **= 9)**				
	No variables with *P* < 0.1			
**Time to recurrence in non-cirrhotic patients (** ***N*** **= 9)**				
	No variables with *P* < 0.1			

Abbreviations: CI, confidence interval; ECOG, Eastern Cooperative Oncology Group; HR, hazard ratio; HVPG, hepatic venous pressure gradient.

Bold values indicate a *P* value < 0.05.

In the overall cohort, the preoperative HVPG level was a significant independent risk factor for poorer TTR (hazard ratio [HR], 1.26 [95% CI, 1.09–1.46]; *P* = 0.002), but not for OS. ROC analysis revealed a HVPG cut-off value of 7.5 mmHg (area under curve [AUC], 0.76 [95% CI, 0.60–0.92]; *P* = 0.007) for reduced TTR (Kaplan–Meier analysis: ≥7.5 mmHg: 17.18 [95% CI, 10.42–23.94] months versus <7.5 mmHg: 43.81 [95% CI, 27.11–60.5] months; *P* = 0.009; see Figure 1). Additional independent risk factors for reduced TTR in the overall cohort were serum creatinine (HR, 1.04 [95% CI, 1.02–1.07]; *P* = 0.002) and size of largest lesion (HR, 1.03 [95% CI, 1.01–1.05]; *P* = 0.004). However, no significant cut-offs were found in ROC analysis (serum creatinine: AUC, 0.46 [95% CI, 0.27–0.65]; *P* = 0.664; size of largest lesion: AUC, 0.57 [95% CI, 0.38–0.76]; *P* = 0.503). There were no significant independent risk factors for 90-day survival or OS in the overall cohort.

**Figure 1:** Kaplan–Meier curves for the determined significant cut-off values for time to recurrence in the overall cohort (a) or overall survival (b) and time to recurrence (c) in patients with cirrhosis after liver resection.

Subgroup analysis in patients with cirrhosis showed HVPG to be an independent risk factor for poorer OS (HR, 1.28 [95% CI, 1.01–1.61]; *P* = 0.041) and TTR (HR, 1.46 [95% CI, 1.14–1.86]; *P* = 0.002). Cut-off values of 8.5 mmHg (AUC, 0.80 [95% CI, 0.56–1.05]; *P* = 0.015) for poorer OS and 7.5 mmHg (AUC, 0.80 [95% CI, 0.63–0.98]); *P* = 0.001) for TTR were identified in ROC analysis. For the determined cut-offs, Kaplan–Meier analysis (Figure 1) demonstrated a significantly reduced OS (≥8.5 mmHg: 44.39 [95% CI, 32.27–56.50] months); <8.5 mmHg (76.84 [95% CI, 68.91–84.77] months; *P* = 0.012) and TTR (≥7.5 mmHg: 20.4 [95% CI, 13.01–27.78] months; <7.5 mmHg: 54.05 [95% CI, 35.9–72.19] months; *P* = 0.007). Serum creatinine and ECOG status at baseline were independent risk factors for reduced TTR in Cox regression for cirrhotic patients, although ROC analysis displayed no significant cut-off values (serum creatinine: AUC, 0.48 [95% CI, 0.26–0.7]; *P* = 0.844; ECOG status: AUC, 0.58 [95% CI, 0.35–0.8]; *P* = 0.513).

In non-cirrhotic patients, no risk factors for OS, TTR, or 90-day survival were demonstrated.

### 3.4 Independent risk factors for postoperative complications and prolonged hospital stay

The logistic regression results for 90-day post-resection complications and prolonged hospital stay are summarised in Table 4. The HVPG level was not associated with post-resection complications in the overall cohort or sub-cohorts. The only significant independent risk factor was total bilirubin at baseline for acute kidney injury in the overall cohort (odds ratio (OR), 1.37 [95% CI, 1.02–1.83]; *P* = 0.036). Patient age was the only other significant parameter in univariable analysis predicting new/worsening ascites (OR, 1.16 [95% CI, 1.02–1.31]; *P* = 0.028). Cut-off values in ROC analysis were a total bilirubin level of 15.5 μmol/L for predicting acute kidney injury (AUC, 0.77 [95% CI, 0.57–0.97]; *P* = 0.007) and a patient age of 62 years (AUC, 0.71 [95% CI, 0.55–0.87]; *P* = 0.011) for new/worsening ascites after resection. In the sub-cohort analysis, no significant independent risk factors for post-resection complications were found.

**Table 4:** Results of univariable and multivariable logistic regression analysis for 90-day post-resection complications and prolonged hospital stay in the overall cohort and patients with or without cirrhosis

Complications	Variables	Univariable logistic regression OR (95% CI)	*P* value	Multivariable logistic regression OR (95% CI)	*P* value
**Overall cohort (** ***N*** **= 38)**					
Prolonged hospital stay					
	ECOG status	9.33 (0.91–95.57)	0.060	10.5 (1.01–108.76)	**0.049**
	UICC stage	2.62 (1.08–6.37)	**0.034**		
Liver dysfunction					
	Total bilirubin	1.24 (0.99–1.55)	0.063		
New/worsening ascites					
	Age	1.16 (1.02–1.31)	**0.028**		
Hospital-acquired pneumonia					
	Total bilirubin	1.21 (0.97–1.50)	0.091		
Acute kidney injury					
	Total bilirubin	1.27 (1.02–1.59)	**0.031**	1.37 (1.02–1.83)	**0.036**
	MELD score	1.29 (0.96–1.74)	0.098		
**Patients with cirrhosis (** ***N*** **= 29)**					
Prolonged hospital stay					
	ECOG status	12.8 (1.15–142.58)	**0.038**	16 (1.38–185.41)	**0.027**
	UICC stage	8.42 (1.18–60.14)	**0.034**		
Liver dysfunction					
	Total bilirubin	1.28 (0.98–1.67)	0.076		
New/worsening ascites					
	Number of lesions	3.26 (0.82–12.92)	0.093		
	Age	1.15 (0.99–1.34)	0.071		
	Average lesion size	1.06 (1.00–1.13)	0.051		
Acute kidney injury					
	Total bilirubin	1.29 (1.00–1.65)	0.050		
**Non-cirrhotic patients (** ***N*** **= 9)**					
	No variables with *P* < 0.1 for any complication				

Abbreviations: CI, confidence interval; ECOG, Eastern Cooperative Oncology Group; MELD, model for end-stage liver disease; OR, odds ratio; UICC, Union for International Cancer Control.

Bold values indicate a *P* value < 0.05.

The median hospital stay length in the overall cohort was nine (range: 4–58) days. The ECOG status was an independent risk for a prolonged hospital stay in the overall cohort (OR, 10.5 [95% CI, 1.01–108.76]; *P* = 0.049) and in patients with cirrhosis (OR, 16 [95% CI, 1.38–185.41]; *P* = 0.027).

## 4 Discussion

In this study, the preoperative HVPG level was a significant independent risk factor for reduced TTR but not OS when considering all HCC patients who received liver resection with curative intent. In the subgroup analysis of patients with cirrhosis, the HVPG was also an independent risk factor for poorer OS. Cut-off values for reduced TTR were 7.5 mmHg in the overall cohort and 8.5 mmHg for poorer OS in cirrhotic patients. When considering only non-cirrhotic patients, HVPG was no risk factor in survival analysis. Furthermore, the HVPG level was no risk factor for 90-day survival, post-resection complications or prolonged hospital stay in any cohort.

Several studies have investigated the impact of preoperative HVPG values on postoperative complications in cirrhotic HCC patients. The reported 90-day mortality after HCC resection in patients with HVPG values of ≥10 mmHg ranges from 0 to 28%, which is in line with the 10% of patients (one out of ten) with an initial HVPG ≥10 mmHg in our study [13,14,17,26,27,28,29]. While some authors found significant differences in 90-day mortality between patients with and without CSPH [17], the majority did not [14,26,27,28,29], including our study. However, it is difficult to compare these results in detail due to differences in baseline characteristics, resection techniques, and study designs. The association of HVPG levels with postoperative ascites, haemorrhage, encephalopathy, or prolonged hospitalisation is also variable in the literature, with cut-off values ranging from >5 to ≥10 mmHg and varying significant findings [13,14,17,26,27,30]. We could not identify the HVPG level as an independent risk factor for any observed postoperative complication in patients with or without cirrhosis and found no differences between patients with and without CSPH. Some studies additionally reported that HVPG values of ≥10 mmHg are associated with postoperative liver dysfunction, decompensation in patients with cirrhosis, or prolonged hospitalisation, which was not the case in our study [13,14,17,26,28,29]. This might result from the small number of patients with CSPH and cirrhosis (*N* = 9 (24%)) in our cohort and, therefore, a low incidence of complications.

Several studies have examined the impact of HVPG measurements on long-term outcomes after HCC resection. Azoulay et al. found 1-/3-year OS rates of 89%/73% and 1-/3-year recurrence-free survival rates of 82%/62% in 79 cirrhotic HCC patients who underwent resection with HVPG values ≥10 mmHg [13]. These results were more favourable compared to our patients with CSPH (1-/3-year OS rates: 90%/58.3%; 1-/3-year recurrence-free rates: 60%/0%). While median MELD scores (8 versus 7 in our study) and Child-Pugh scores (*N* = 78 (99%) versus *N* = 36 (95%) with Child-Pugh A in our study) were comparable, significantly more patients with microvascular (*N* = 25 (32%) versus *N* = 27 (71%) in our study) and macrovascular tumour invasion (*N* = 3 (4%) versus *N* = 10 (26%) in our study) at time of resection might have led to a worse overall outcome in our analysis.

Llovet et al. found a significantly lower median OS in 43 cirrhotic patients with CSPH undergoing HCC resection after HVPG measurement, with 69 months in patients with an HVPG ≥10 mmHg versus 80 months in patients with <10 mmHg [31]. These results are comparable to the cut-off value of 8.5 mmHg found in our study to predict a worse OS in cirrhotic patients (≥8.5 mmHg: 44.39 months; <8.5 mmHg: 76.84 months). In contrast, other authors reported no significant associations between the HVPG and OS. Cucchetti et al. analysed 70 HCC patients with and without cirrhosis after HCC resection and found non-significant differences in 1-/3-year OS rates with 100%/100% in patients with a baseline HVPG <10 mmHg and 97.1%/79.4% in patients with HVPG levels ≥10 mmHg [14]. A possible explanation could be the combined analysis of patients with (*N* = 46 (66%)) and without cirrhosis (*N* = 24 (34%)) without comparing the subgroups. While patients with CSPH (of which nine (90%) out of ten patients had cirrhosis) in our cohort had lower averaged 1-/3-year OS rates of 90%/58.3%, patients without CSPH at baseline had comparable OS rates of 92.9%/82.1%. However, a detailed comparison of the cohort characteristics is not possible due to imbalances in sample size and the lack of pathological information provided.

Furthermore, Silva et al. showed that the HVPG level was no risk factor for poorer OS in univariable or multivariable analysis of 22 Child-Pugh A cirrhosis patients with resected HCC of a single nodule up to 5 cm [32]. In contrast, our study found a significant impact of HVPG on OS in cirrhotic patients, of which 27 (93%) had a Child-Pugh A score, although resection was performed in the presence of up to four lesions and a tumour size of up to 110 mm. Other results favouring the HCC resection in Child-Pugh A patients despite CSPH were described by Cortese and Tellado analysing 42 matched HCC patients with Child-Pugh A cirrhosis undergoing hepatic resection with or without CSPH, respectively, reporting no significant differences in 1-/3-year OS rates (CSPH: 85.7%/64.0%; non-CSPH: 92.9%/70.1%; *P* = 0.604) or disease-free survival rates (CSPH: 61.3%/44.4%; non-CSPH: 59.5%/29.5%; *P* = 0.296) [29]. Although 1-/3-year OS rates (CSPH: 90%/58.3%; non-CSPH: 92.9%/82.1%; *P* = 0.146) were comparable in our study, 1-/3-year recurrence-free rates (CSPH: 60%/0%; non-CSPH: 72.1%/42.2%; *P* = 0.048) were significantly reduced in patients with CSPH. Given that the patient characteristics between our studies – although again limited comparable – do not considerably differ, the analysis of a smaller cohort of ten (26%) CSPH patients may have resulted in sample bias, contributing to the fact that no CSPH patient remained disease-free after three years post-surgery in our study.

In summary, varying associations between pre-resection HVPG levels and long-term outcomes are reported in the literature, making it difficult to recommend pre-resection HVPG measurement in patients with HCC per se. However, in HCC patients with suspected liver cirrhosis or patients who are borderline surgical candidates, HVPG measurement could be performed simultaneously with a transjugular liver biopsy as an additional marker of disease extent to assist in the decision for or against liver resection. Moreover, combining HVPG measurement with liver biopsy could be particularly useful, as our study intends that abnormal HVPG values should not be considered as an absolute contraindication for liver resection, and a comprehensive assessment of other risk factors such as underlying cirrhosis is essential for an adequate evaluation of potential surgical candidates. Larger, prospective studies are needed to further validate the benefit of HVPG measurement before liver resection.

### 4.1 Limitations

Our study has limitations. The relatively small sample size might have led to sample bias, especially in the smaller non-cirrhotic or CSPH group. Transplantation remains the preferred option for cirrhotic patients within the criteria. Moreover, our current practice favours ablative therapies over liver resection for borderline surgical candidates. Since we only perform HVPG measurements when liver cirrhosis is suspected clinically or by imaging, and the majority were subsequently classified as cirrhotic, thus ultimately limiting the statistical power of our analysis. Due to the retrospective nature of this study, we could not assess for missing information in the medical reports. Therefore, we could not identify the specific catheters used in 31 out of 38 patients and were unable to compare HVPG levels and outcomes between patients with balloon occlusion and conventional catheter measurements. However, both techniques have been recognised in the literature, were performed with at least three repeated measurements, and were assessed in combination with the inferior vena cava and right atrial pressures as internal reference [33,34]. Notably, we have adopted the use of balloon occlusion catheters only to standardise the HVPG measurement at our centre since the completion of this study, which is now also the recommended approach in the most recently published Baveno VII Consensus Workshop to reduce random errors in WHVP measurement [35]. Finally, it should be noted that the FHVP level is affected by the catheter tip position and vein morphology, which may result in varying results, especially among different operators [36]. However, all investigators in our centre followed the same standard operating procedure.

## 5 Conclusions

Our results indicate that the preoperative HVPG level in cirrhotic patients with HCC undergoing liver resection has a significant clinical impact on the long-term outcome with poorer OS and TTR from HVPG levels of 8.5 and 7.5 mmHg, respectively, while the occurrence of postoperative complications appears to be independent of the HVPG.
